# Effect of Programmed Comprehensive Nursing for Postoperative Delirium in Intensive Care Unit Patients

This article has been retracted.

**DOI:** 10.1155/2022/1227659

**Published:** 2022-05-11

**Authors:** Juanjuan Liao, Chuanran Kui, Yangchun Zhou, Li Huang, Dandan Zuo, Yuqin Huang, Ruihong Pan

**Affiliations:** ^1^Department of Intensive Care Unit, Suizhou Hospital, Hubei University of Medicine, Suizhou, Hubei Province, China; ^2^Department of Nursing, Suizhou Hospital, Hubei University of Medicine, Suizhou, Hubei Province, China

## Abstract

**Background:**

This study is to evaluate the effect of programmed comprehensive nursing for postoperative delirium in intensive care unit (ICU) patients.

**Methods:**

A total of 90 cases of ICU surgery patients admitted to our hospital from July 2019 to July 2020 were recruited and assigned via the random number table method (1 : 1) to receive either conventional nursing (control group) or programmed comprehensive nursing (experimental group). The delirium assessment method was used to record the incidence of delirium events at different time points after the intervention. Outcome measures included delirium events, the Visual Analogue Scale (VAS) scores, the Pittsburgh sleep quality index (PSQI) scores, the activities of daily living (ADL) scale scores, nursing satisfaction, and total nursing efficiency.

**Results:**

Programmed comprehensive nursing was associated with significantly better nursing satisfaction, ADL scores, VAS scores, PSQI scores, and nursing efficiency than conventional nursing (all *P* < 0.05). Programmed comprehensive nursing resulted in a significantly lower incidence of postoperative delirium than conventional nursing (*P* < 0.05).

**Conclusion:**

The application of programmed comprehensive nursing for postoperative delirium in ICU patients shows a promising efficiency, effectively alleviates the clinical symptoms of patients, and optimizes various clinical indicators of patients; hence, it is worthy of further application and promotion.

## 1. Introduction

The severe condition and symptoms of ICU patients are associated with multiple postoperative complications, among which postoperative delirium is common, especially among elderly people, with high mortality. Its manifestations include restlessness, loss of orientation, confusion, paresthesia, and speech disorder. Its etiology is related to a variety of infectious diseases and neurological diseases. Relevant studies have shown that postoperative delirium is prone to cause multiple complications, such as respiratory failure, lung infection, and brain-heart syndrome, which seriously threatens the patients' health and impairs their quality of life [1–4]. In recent years, nursing measures for postoperative delirium exerts a tremendous influence on the academia. Most scholars believe that adequate nursing measures can effectively reduce the incidence of postoperative delirium events in patients. Furthermore, the desire for better nursing care is growing among people who have shown dissatisfaction with conventional nursing. Programmed comprehensive nursing, a patient-oriented nursing mode, is widely used in clinical nursing and has achieved significant nursing effects compared to conventional nursing. Therefore, this study is to evaluate the effect of programmed nursing for postoperative delirium on ICU patients.

## 2. Materials and Methods

### 2.1. General Information

A total of 90 cases of ICU surgery patients admitted to our hospital from July 2019 to July 2020 were recruited and divided into a control group (*n* = 45 cases) and an experimental group (*n* = 45 cases) according to the random number table method. This study was certified by the Ethics Committee of Suizhou Hospital, Hubei University of Medicine, with ethics certificate number 2018-11-11.

### 2.2. Inclusion Criteria

Inclusion criteria were as follows: (1) all patients met the diagnostic criteria for postoperative delirium; (2) patients with complete clinical data were included; (3) this study was approved by our hospital ethics committee. The patients and their families signed an informed consent form after being fully informed of the purpose and the process of the study.

### 2.3. Exclusion Criteria

Exclusion criteria were as follows: (1) the patients with mental and other cognitive disorders; (2) patients with incomplete clinical data; (3) patients who did not cooperate with the research.

### 2.4. Methods

The control group used conventional nursing.

The experimental group received programmed comprehensive nursing on the basis of conventional nursing, and the specific measures were as follows: (1) Due to the limited mobility and decreased ability after surgery, the patients are prone to negative emotions such as anxiety, irritability, and depression. Therefore, medical staff should provide psychological counseling to the patients in time to eliminate their negative emotions. The patients were also given dietary guidance and health education. In addition, the staff should actively communicate with patients and satisfy the requirements of patients in a timely manner to establish a friendly nurse-patient relationship. For patients with communication difficulties, nursing staff should provide appropriate encouragement and guidance to reduce their psychological pressure. (2) Most patients might refuse to take analgesics and endure postoperative pain due to their worries of drug dependency, which would easily lead to hysteria-like hallucinations and delirium [5–7]. Moreover, these patients had difficulty in communication before surgery and poor postoperative compliance. Thus, medical staff should assess the patient's pain in a timely manner and adopt targeted treatment measures and psychological counseling to help them reduce psychological resistance to analgesics. (3) Postoperative delirium is also related to hypoxemia. To prevent delirium, low-flow oxygen inhalation to the patients was necessitated, with the oxygen flow adjusted according to the actual condition to ensure a stable aerobic state for the brain and avoid delirium events. (4) If the patient had delusions or sleep disturbance, the doctor should be notified in time and effective treatment measures should be taken to lower the incidence of delirium in the patients. (5) The poor sleep quality of patients is attributed to excessive worry about their conditions. Therefore, medical staff should help patients arrange a reasonable sleeping schedule, and for patients who have difficulty in sleeping, drugs could be provided when necessary.

### 2.5. Indicator Observation

The “Patient Clinical Satisfaction Questionnaire” [8] prepared by the department was used to investigate the satisfaction of patients after nursing. The questionnaire is divided into three scores: satisfied, basically satisfied, and dissatisfied. Total satisfaction = satisfied + basically satisfied.

The treatment effect of the two groups of patients was observed. Markedly effective was defined as clinical symptoms have been significantly alleviated. Effective was defined as clinical symptoms have been alleviated. Ineffective was defined as the clinical symptoms have not been alleviated or even worsened.

The total incidence of delirium in the two groups was compared. The time periods of 1 d, 3 d, and 5 d after the operation of the two groups of patients were set as T0, T1, and T2, and the incidence of delirium at different time points in the two groups was recorded.

The “Visual Analogue Scale (VAS)” [9] was used to evaluate the pain of the patients after the operation. The total score on the scale was 10 points. The higher the score, the more severe the pain of the patient.

The “Pittsburgh Sleep Quality Index (PSQI) scale” [10] was used to evaluate the patient's sleep quality before and after the intervention. The total score on the scale was 15 points. The higher the score, the worse the patient's sleep quality.

The “activities of daily living (ADL) scale” [11] was used to evaluate the patient's self-care ability recovery status. The score was 0–100 points. The higher the score, the better the recovery of the patient's self-care ability.

### 2.6. Statistical Methods

The experimental data were statistically analyzed and processed by SPSS21.0 software, and GraphPad Prism 7 (GraphPad Software, San Diego, USA) was used to plot graphics of this data. Count data were expressed as (*n*(%)) and processed using the *x*^2^ test, and measurement data were represented by $\left(\bar{x}\pm s\right)$ and analyzed using the *t*-test. When *P* < 0.05, the difference was considered statistically significant.

## 3. Results

### 3.1. General Information Comparison

The two groups did not show a great disparity in terms of age, gender, BMI, education level, smoking, drinking, and the place of residence (*P* > 0.05), as shown in Table 1.

### 3.2. Comparison of Nursing Satisfaction between the Two Groups

Programmed comprehensive nursing was associated with significantly better nursing satisfaction than conventional nursing (*P* < 0.05), as shown in Figure 1.

### 3.3. Comparison of ADL Scores and VAS Scores between the Two Groups

The ADL scores of the two groups of patients after intervention were significantly elevated (*P* < 0.05), with higher ADL scores of patients in the experimental group than those of the control group (*P* > 0.05) (Figures 2(a) and 2(b)).

### 3.4. Comparison of PSQI Scores between the Two Groups

There was no significant difference in PSQI scores between the two groups before intervention (*P* > 0.05). Programmed comprehensive nursing was associated with significantly higher ADL scores than conventional nursing (*P* < 0.05) (Table 2).

### 3.5. Comparison of Nursing Efficiency of the Two Groups of Patients

The total efficiency of nursing care in the experimental group was 97.78%, which was markedly higher than that of 82.22% in the control group (*P* < 0.05), as shown in Figure 3.

### 3.6. Comparison of the Incidence of Postoperative Delirium between the Two Groups

Programmed comprehensive nursing resulted in a significantly lower incidence of postoperative delirium than conventional nursing (*P* < 0.05) (Table 3).

## 4. Discussion

To date, the pathogenesis of delirium has not yet been clarified. Risk factors for delirium include the metabolism of the brain, severe emergency response, sleep disorders, brain geological system, and toxins. Delirium is a frequent postoperative complication among ICU patients. Moreover, the long-term state of hypoperfusion in ICU patients after surgery and the reduced cardiac output may increase the incidence of delirium [12–15]. As one of the acute brain dysfunctions, delirium is characterized by clinical symptoms of fluctuating thinking disorder and disturbance of consciousness, such as delusion and hallucination. In addition, the patients suffer a poor memory and in severe cases, environmental disorientation as a result of sleep-wake rhythm disorder. Elderly people are more susceptible to the disease as their body functions are severely degraded, and the level of the pancreas decreases, thus leading to an increase of norepinephrine and poor memory after surgery. Furthermore, the function of the regulatory system will be weakened, and they will become excessively sensitive to external stimuli, which is one of the main reasons for delirium. The patient's body intolerance to severe postoperative pain will directly compromise the patient's body function, which may consequently trigger delirium [16–19]. After surgery, hypoxemia in ICU patients may cause disorientation, hallucinations, irritability, and other negative emotions, with which patients are prone to self-injury, accidental extubation, and falling from bed. Therefore, it is indispensable to conduct a risk assessment promptly and take effective protective measures to ensure the safety of patients. In recent years, the desire for better nursing care is growing among people. Programmed comprehensive nursing, being widely used in clinical nursing, has achieved significant nursing effects. It is patient-centered, meets patients' psychological demands, provides patients with a comfortable hospitalization environment, improves patients' nursing satisfaction and quality of care, and promotes patients' speedy recovery [20–23]. The results of this study showed that the total efficiency rate of nursing care in the experimental group was 97.78%, which was significantly better than the rate of 82.22% in the control group (*P* < 0.05), which was consistent with the research results by Wang et al. Their research results stated that “the experimental group obtained a higher effective rate of 96.45%, in comparison with the rate of 81.34% in the control group (*P* < 0.05)”, which substantially proved that the application of programmed comprehensive nursing to ICU patients can significantly alleviate the clinical symptoms of patients, strengthen their quality of care, enhance nursing satisfaction, promote postoperative recovery, and ensure a promising nursing effect.

The incidence of postoperative delirium is directly proportional to age. It has been shown that the incidence of postoperative delirium is significantly higher in patients ≥70 years of age, mainly due to decreased cerebral blood supply in the elderly, sensitivity to intraoperatively induced hypoxia, and poor pulmonary compliance, all of whom are not disconnected from ventilator-assisted breathing after surgery. They are highly sensitive to mild hypoxia, and premature extubation may lead to a decrease in the central nervous system transmitter acetylcholine, resulting in the development of delirium. Programmed comprehensive care can mitigate delirium risk factors such as surgical pain, environmental stress, hypoproteinemia, medications, and infection. The key to preventing and treating postoperative ICU delirium lies in good preoperative preparation and careful postoperative care. Nursing interventions, especially psychological care, play an important role in reducing the incidence of postoperative delirium, which is conducive to reducing the incidence of complications and improving recovery outcomes. The core of TCM nursing is evidence-based nursing care throughout the entire care process and requires close observation of changes in the condition of elderly patients in the ICU, implementation of routine nursing measures such as routine vital sign detection, tracheal intubation, and intravenous placement. Moreover, in TCM care, the risk factors for postoperative delirium are assessed, and the patients are actively treated with their primary diseases to prevent postoperative infections, cardiovascular and cerebrovascular diseases, and other complications and maintain electrolyte balance. In addition, drugs that are less irritating to patients, especially traditional Chinese medicine preparations with unique efficacy, respiratory support therapy, diet modification, and improvement of the ICU environment are applied. In the acute phase of postoperative delirium, sedation therapy is actively given to control the psychiatric symptoms.

Ischemic damage to the brain is commonly considered the cause of delirium. Associated with delirium are higher concentrations of S-100*β* protein, a protein that is abundant in astrocytes and Schwann cells and is found in organs such as the brain, heart, skeletal muscle, and kidneys. However, elevated concentrations of S-100*β* protein are insufficient to identify brain damage and disruption of the blood-brain barrier. Dopamine is an important neurotransmitter for motor function, attention, and cognitive performance. Dopamine receptors (D1 to D5) can be divided into 2 families. The activity of D1-family (D1 and D5 receptors) receptors increases acetylcholine cachexia, whereas the activity of D2, D3, and D4 receptors decreases acetylcholine cachexia. The number of D1 and D2 receptors decreases with age, so the probability of delirium increases in older individuals. Dopamine drug intoxication, such as levodopa, may trigger hyperactivity-type delirium due to the role of acetylcholine and metabolic factors in the synthesis of dopamine. Proinflammatory cytokines are produced in the periphery and interact with the brain, especially interleukin-1*β* (IL-1*β*), tumor necrosis factor I only (TNF-*α*), and IL-6. Peripheral-specific cytokine signals can be transmitted to the brain by several extant mechanisms into direct neural pathways via vagal afferents and transported through the blood-brain barrier or into the brain via periventricular areas. These cytokines induce the production of inflammatory cytokines by small glial cells in the brain. In a rat model of surgically induced cognitive decline, TNF induces IL-1 synthesis in the brain and peripheral blockade of TNF-*α* reduces IL-1 production, which can reduce the occurrence of neuroinflammation as well as the decline in cognitive function. The aging process can be seen as a primitive stimulation of neuroglia, which is restimulated by peripheral signal-mediated inflammatory responses and some of the stimulated neuroglia release excessive amounts of proinflammatory response cytokines, which explains the rather minor triggers that predispose the elderly to delirium. Elevated concentrations of C-reactive protein (CRP) are associated with the development of delirium, but it has also been suggested that CRP is not associated with cognitive dysfunction but with depression. Programmed comprehensive care in patients with postoperative delirium in the ICU is effective in alleviating the patient's inflammatory response, optimizing all clinical indicators, and reducing the incidence of delirium.

## 5. Conclusion

The application of programmed comprehensive nursing for postoperative delirium in ICU patients shows a promising effect, effectively alleviates the clinical symptoms of patients, and ameliorates various clinical indicators of patients; hence, it is worthy of further application and promotion.

## Figures and Tables

**Figure 1:** Comparison of satisfaction between the two groups (*n* (%)). (a) The expression of the nursing effect on the experimental group. (b) The expression of the nursing effect on the control group. The satisfied rate of the experimental group was 71.11% (32/45), the basically satisfied rate was 22.22% (10/45), the dissatisfied rate was 6.67% (3/45), and the overall satisfaction rate was 93.33% (42/45); moreover, the satisfied rate of the control group was 44.44% (20/45), the basically satisfied rate was 28.89% (13/45), the dissatisfied rate was 26.67% (12/45), and the overall satisfaction rate was 73.33% (33/45). There was a significant difference between the two groups of patients after nursing (*x*^2^ = 6.480, *P*=0.011).

**Figure 2:** Comparison of ADL scores and VAS scores between the two groups of patients $\left(\bar{x}\pm s\right)$. (a)The abscissa represents the preintervention and postintervention, and the ordinate represents the ADL score and points. The ADL scores of patients in the experimental group before and after intervention were (77.42 ± 6.93) points and (88.69 ± 7.93) points, respectively, and the ADL scores of the control group before and after intervention were (77.15 ± 6.58) points and (83.12 ± 7.21) points, respectively, where the symbol ^*∗*^ indicates that there was a significant difference in the ADL scores of the experimental group before and after intervention (*t* = 7.179, *P* < 0.05); the symbol ^*∗∗*^ indicates that there was a significant difference in the ADL scores of the control group before and after intervention (*t* = 4.103, *P* < 0.05); and the symbol ^*∗∗∗*^ indicates that there was a significant difference in the ADL scores of the two groups before and after intervention (*t* = 3.486, *P* < 0.05). (b) The abscissa represents the experimental group and control group after intervention, and the ordinate represents the VAS score and points. The VAS scores of the experimental group before and after intervention were (7.23 ± 1.35) points and (3.02 ± 0.59) points, respectively, and the VAS scores of the control group before and after intervention were (7.11 ± 1.42) points and (5.87 ± 1.13) points, respectively; the symbol ^*∗*^ indicates that the VAS scores of patients in the experimental group before and after intervention were significantly different (*t* = 19.169, *P* < 0.05); the symbol ^*∗∗*^ indicates that there was a significant difference in the VAS scores of the control group before and after intervention (*t* = 4.584, *P* < 0.05); the symbol ^*∗∗∗*^indicates that the VAS scores of the two groups of patients after intervention were significantly different (*t* = 14.998, *P* < 0.05).

**Figure 3:** Comparison of nursing effects between the two groups (*n* (%)). (a) The expression of the nursing effect in the experimental group. (b) The expression of the nursing effect in the control group. In the experimental group, the markedly effective rate was 68.89% (31/45), the effective rate was 28.89% (13/45), the ineffective rate was 2.22% (1/45), and the total effective rate was 97.78% (44/45), and in the control group, the markedly effective rate was 51.11% (21/45), the effective rate was 35.56% (16/45), the ineffective rate was 17.78% (8/45), and the total effective rate was 82.22% (37/45). There were significant differences between the two groups of patients after intervention (*x*^2^ = 6.049, *P* < 0.05).

**Table 1:** Comparison of general information between the two groups of patients (*n* (%)).

	Experimental group (*n* = 45)	Control group (*n* = 45)	X^2^ or t	*P*
Gender			0.044	0.833
Male	21 (46.67)	22 (48.89)		
Female	24 (53.33)	23 (51.11)		
Age (years)			0.239	0.811
	40.89 ± 3.86	41.08 ± 3.67		
BMI (kg/m^2^)			0.563	0.574
	26.14 ± 1.67	25.93 ± 1.86		
Education level				
Primary school or below	9 (20.00)	8 (17.78)	0.072	0.788
Middle school	14 (31.11)	16 (35.56)	0.200	0.655
High school and technical secondary school	15 (33.33)	16 (35.56)	0.049	0.824
Junior college and above	7 (15.56)	5 (11.11)	0.384	0.535
Smoking			0.049	0.824
Yes	30 (66.67)	29 (64.44)		
No	15 (33.33)	16 (35.56)		
Drinking			0.177	0.673
Yes	22 (48.89)	24 (53.33)		
No	23 (51.11)	21 (46.67)		
Place of residence			0.182	0.670
Urban	27 (60.00)	25 (55.56)		
Rural	18 (40.00)	20 (44.44)		

**Table 2:** Comparison of PSQI scores between the two groups $\left(\bar{x}\pm s\right)$.

Groups	n	Before intervention	After intervention
Experimental group	45	11.27 ± 3.71	3.28 ± 1.12
Control group	45	11.33 ± 3.66	6.88 ± 1.31
*x* ^2^		0.077	9.923
*P* value		＞0.05	<0.05

**Table 3:** Comparison of the incidence of postoperative delirium between the two groups (*n* (%)).

Groups	n	*T*_0_	*T*_1_	*T*_2_	Total incidence of delirium
Experimental group	45	4.44% (2/45)	4.44% (2/45)	0.00% (0/45)	8.89% (4/45)
Control group	45	11.11% (5/45)	11.11% (5/45)	8.89% (4/45)	31.11% (14/45)
*x* ^2^					6.944
*P*					*P* < 0.05

## Data Availability

The datasets used during the present study are available from the corresponding author upon reasonable request.
